The article "Lycium barbarum polysaccharides inhibit proliferation and migration of bladder cancer cell lines BIU87 by suppressing Pi3K/AKT pathway" was retracted in 2026. Reasons: plagiarized images; duplicated images; overlap with other authors' work; original data or images not available.

# Lycium barbarum polysaccharides inhibit proliferation and migration of bladder cancer cell lines BIU87 by suppressing Pi3K/AKT pathway

**DOI:** 10.18632/oncotarget.13963

**Published:** 2016-12-15

**Authors:** Xian-Jun Zhang, Hong-Yuan Yu, Yong-jian Cai, Mang Ke

**Affiliations:** ^1^ Department of Urology, Taizhou Hospital of Zhejiang Province, Wenzhou Medical University, Linhai, Zhejiang Province, PR China

**Keywords:** lycium barbarum polysaccharides, bladder cancer, Pi3K/AKT, proliferation, migration

## Abstract

The aim of this study was to verify whether *Lycium barbarum polysaccharides* inhibits proliferation and migration of BIU87 cells through Pi3K/AKT pathway. Different concentrations of *Lycium barbarum polysaccharides* were used to incubate with BIU87cells. LY-294002 and IGF-1 were used to inhibit and activate Pi3K/AKT pathway respectively. MTT were used to investigate the proliferation of BIU87cells. Transwell chambers and wound healing were used to test the migratory ability of BIU87cells. Western blotting were used to investigate the expressions of P21,P27,MMP-2, MMP-9, AKT and p-AKT in BIU87cells. Compared with the control group, the proliferation and migration of BIU87cells and the expression of p-AKT were significantly decreased in the study group; the inhibitory effect of the downregulation of p-AKT by LY-294002on the induction of BIU87cells proliferation and migration was identical to that of *Lycium barbarum polysaccharides*; upregulation of p-AKT by IGF-1 reversed the *Lycium barbarum polysaccharides*-induced inhibition of BIU87cells dedifferentiation. In conclusion, LBP inhibits the proliferation and migration of BIU87 cells by suppressing Pi3K/AKT signaling pathway.

## INTRODUCTION

Bladder cancer (BC), is among the fifth most common malignancies in the world [1]. The majority of BC is represented by urothelial carcinoma (UC), or named transitional cell carcinoma (TCC), while squamous and adenocarcinomas are diffused in a small percentage [1]. Although BC is considered to be responsive to the chemotherapy regiments, only few patients respond to single-agent therapy. Because of this, the finding of innovative anti-cancer combinations and new anti-neoplastic drugs is necessary. At present, many researchers are committed to antineoplastic drugs with high activity and low toxicity from nature. Traditional Chinese herbs, with anticancer properties, have drawn a great deal of attention in recent years.

*Lycium barbarum polysaccharides* (LBP), is the major functional component of the fruit of *L. barbarum* (comprising 5%–8% of *L. barbarum fruits*), which is a well-known Chinese herb. Its molecular weight ranges from 24 kDa to 241 kDa and consists of a complex mixture of highly branched and only partly characterized polysaccharides and proteoglycans. LBP shows antitumor activities against various types of cancer cells and inhibit tumor growth in nude mice through induction of apoptosis and cell cycle arrest [2–4]. Mang et al reported that LBP could inhibit the growth of human bladder carcinoma cell line BIU87 and induce BIU87 apoptosis [3]. However, the mechanism of LBP inducing apoptosis of BIU87 cells has yet been unclear.

The article "Lycium barbarum polysaccharides inhibit proliferation and migration of bladder cancer cell lines BIU87 by suppressing Pi3K/AKT pathway" was retracted in 2026. Reasons: plagiarized images; duplicated images; overlap with other authors' work; original data or images not available.

The PI3K/AKT signaling is a critical pathway in cell proliferation, survival, neovascularization and tumor growth [5–6]. As a bridge molecule combining extracellular signal and response effector of cells, PI3K acts on the downstream signaling molecules under the influence of a series of bypass or upstream signaling molecules, and play a very important role in regulating cell apoptosis. Akt/PKB is an important downstream target kinase of PI3K signaling pathway. Activated Akt can inhibit the release of cytochrome c and apoptosis factor, thereby inhibiting apoptosis, and promote the growth of cancer cells. Researches about PI3K/AKT signaling pathway in prostate cancer, colorectal cancer and lung cancer have been widely reported [7–9]. However, the relationship between the PI3K/AKT signaling pathway and proliferation and migration of bladder cancer cells has not yet been reported. The present study was designed to study whether PI3K/AKT signaling pathway can promote the proliferation and migration of BIU87 cells, whether LBP can inhibit the proliferation and migration of BIU87cells by inhibiting PI3k/AKT pathway.

## RESULTS

### LBP can inhibit the proliferation and migration of BIU 87cells

MTT results showed that under various culture conditions, compared to the control group, OD value of LBP groups was significantly lower (all *P* < 0.05), presenting dose/effect and time/effect relationship (Figure 1A). WB results showed that, compared to the control group,P21, P27 expression of LBP group significantly increased according to the WB gray analysis (*p* < 0.05), and positively correlated with the dose of LBP (Figure 1B). Obviously, the results of MTT and WB both suggested LBP could inhibit the proliferation of BIU87cells. The results of transwell assay and wound healing showed that compared with the control group, BIU87 cell migration was significantly reduced (*P* < 0.05), and positively correlated with the dose of LBP (Figure 1C). The results of protein immunoblotting showed that compared to the control group, the expression of MMP-2 and MMP-9 in LBP groups were both significantly reduced (both *P* < 0.05) and was positively correlated with the dose of LBP (Figure 1D). The results of transwell assay and wound healing both suggested LBP could inhibit the migration of BIU87cells.

The article "Lycium barbarum polysaccharides inhibit proliferation and migration of bladder cancer cell lines BIU87 by suppressing Pi3K/AKT pathway" was retracted in 2026. Reasons: plagiarized images; duplicated images; overlap with other authors' work; original data or images not available.

**Figure 1:** LBP can inhibit the proliferation and migration of BIU 87cells (**A**) Effects of LBP on the proliferation of BIU87cells at different times; (**B**) Effects of LBP on the BIU87cells expression of P21 and P27; (**C**) the upper photo shows the migration of BIU87cells 48 hours after being scratched (×100), while the below photo shows DAPI staining pattern of BIU87cells migrating to lower chamber 48 hours after transwell (×200); (**D**) Western blot analysis of MMP-2 and MMP-9 expression in BIU87 cells of each group.

### LBP inhibit activation of PI3K/AKT pathway

As we can see in Figure 2, AKT expression of BIU87 cells between each group was not significantly different (*P* > 0.05). Phosphorylation of Akt is characteristic of PI3K activation. Compared to the Control group, the expression of p-AKT of BIU 87 cells in LBP groups were significantly reduced (*P* < 0.05), was positively correlated with the dose of LBP.

**Figure 2:** Western blot analysis of AKT and p-AKT expression in BIU87 cells of each group

### LBP inhibits the proliferation and migration of BIU87cells by inhibiting PI3k/AKT pathway

LBP concentration in subsequent trials were all 800 μg /ml as the optimum concentration. LY-294002 is a specific inhibitor of Pi3k and can significantly inhibit the expression of p-AKT. After the addition of 20 mmol/L LY-294002, proliferation and migration of BIU 87 cells was significantly decreased; proliferation and migration of BIU87 cells have no significant difference between LBP + LY-294002 group and LBP group (all *P* > 0.05) (Figure 3A, and 3C).

**Figure 3:** LBP inhibits the proliferation and migration of BIU87cells by inhibiting Pi3k/AKT pathway (**A**) Effects of LBP and LY-294002 on the proliferation of BIU87cells at different times by MTT analysis. (**B**) The migration of BIU87 cells under the intervention of different conditions in the wound healing assay and transwell assay. (**C**) Effects of LBP and LY-294002on the BIU87 cells’ expression of AKT and p-AKT by WB analysis.

IGF-1, as agonists of Pi3k , can activate Pi3K and increased expression of p-AKT. When 3 ng/ml IGF-1 was added to cell culture medium, the inhibition effect of LBP on proliferation and migration of BIU87 cells was reversed. The proliferation and migration of BIU87 cells increased significantly (Figure 4A, and 4C).

**Figure 4:** Effects of LBP and IGF-1 on the proliferation and migration of BIU87 cells and the expression of p-AKT (**A**) Effects of LBP and IGF-1 on the proliferation of BIU87 cells at different times; (**B**) The migration of BIU87 cells under the intervention of different conditions in the wound healing assay and transwell assay; (**C**) Effects of LBP and IGF-1on the BIU87 cells’ expression of AKT and p-AKT by WB analysis.

The article "Lycium barbarum polysaccharides inhibit proliferation and migration of bladder cancer cell lines BIU87 by suppressing Pi3K/AKT pathway" was retracted in 2026. Reasons: plagiarized images; duplicated images; overlap with other authors' work; original data or images not available.

## DISCUSSION

Proliferation, invasion and metastasis are the basic biological characteristics of malignant tumors. This is not only associated with the enhanced invasiveness and the decrease adhesion of tumor cells, but also is closely related to tumor angiogenesis, the extracellular matrix degradation and interstitial remodeling [10]. Thus, the inhibition of tumor cell proliferation, invasion and migration is very important for cancer therapy. Although radical cystectomy with chemotherapy has been applied for treating BC patients as the standard clinical administration and exerted efficient benefits, recurrence and metastasis take place frequently [11]. To prevent recurrence and progression, intravesical chemotherapy or immunosuppressive agents have been widely used after radical cystectomy [12]. However, these supplemental methods are largely restricted with various degrees of side effects such as bone marrow suppression, allergic reactions and etc [13]. Thus, there is an unmet demand to develop safe and effective administration strategy for treating BC.

Cancer is a kind of disease with multiple etiologies and multistage processes. However, using non-toxic natural substances to reduce the carcinogenic effect has gradually become a strategy. Researchers have also recently focused on using such agents against cancer cells to induce apoptosis, which represents a programmed self-killing mechanism that involves extrinsic and intrinsic pathways [14]. It is reported that the ethanol extract of pomegranate fruits [15], EGCg [16], resveratrol, grape seed extract [17], and the green tea catechin all could induce the apoptosis of bladder cancer cells [18]. Here, we focused on another active component of lycium barbarum, LBP, which has shown *in vitro* inhibitory effects on many cancer cell lines. Lycium barbarum is a well-known traditional Chinese herbal medicine which has multiple pharmacological and biological functions including neuroprotection [19–20] , antioxidant [21] anti-aging [22],cytoprotection [23] and immuno-odulating [24]. Based on the antioxidant and antiapoptosis activity of LBP, many studies have demonstrated that LBP has anticancer effect in various malignant tumors. Chen et al [25] investigated the putative synergistic immunotherapeutic roles of LBP and IFNα2b against renal cell carcinoma (RCC) *in vitro* and *in vivo*, and the results suggested that the combination of LBP and IFNα2b is likely to be more effective in treating murine RCC compared with the less pronounced immunotherapeutic effects of administering IFN-α2b alone. Zhang et al [26] found that LBP could block human hepatoma SMMC-7721 cells at the G0/G1 and S phases with an inhibition ratio of 45.13%, showing that LBP can be provided as a potential chemotherapeutic agent drug to treat cancer. However, currently researches on the mechanism of anti-tumor effects of LBP are rare.

The article "Lycium barbarum polysaccharides inhibit proliferation and migration of bladder cancer cell lines BIU87 by suppressing Pi3K/AKT pathway" was retracted in 2026. Reasons: plagiarized images; duplicated images; overlap with other authors' work; original data or images not available.

PI3K/AKT pathways is one of signal transduction pathways most closely correlated with cell proliferation and apoptosis. Abnormal activation of PI3K /AKT signaling pathway induces abnormal cell proliferation and differentiation and promotes tumor cell growth. Phosphorylation of AKT generates p-AKT, which can further activate the mTOR pathway, increase the expression of p-mTOR and p-70S6K, and ultimately increase the proliferation and migration of tumor cells. This study found that LBP can inhibit the proliferation and migration of BIU87 cells and reduce the expression of p-AKT. Then we used LY-294002 which is specific inhibitor of Pi3K to pretreatment BIU87 cells and found LY-294002 can inhibit the expression of p-AKT and inhibit the proliferation and migration of BIU87 cells. In addition, IGF-1, as an agonist of Pi3K, was used to pretreatment BIU87 cells. We found IGF-1 can significantly increase the expression of p-AKT, and reverse the inhibition effect of LBP on the proliferation and migration of BIU87. The results finally certified LBP could inhibit the proliferation and migration of BIU87 cells by suppressing PI3K/AKT pathway.

In conclusion, the results suggested that LBP inhibits the proliferation and migration of BIU87 cells by, at least partly, repressing PI3k/AKT pathway. Therefore, LBP may prove beneficial as a therapeutic strategy for bladder cancer treatment.

## MATERIALS AND METHODS

### Experiment reagent

Lycium barbarum polysaccharides was purchased from Xi’an SenRan Biological Engineering Co., Ltd. (Shaanxi, China). The batch number was 20081201, and the content > 30%. Experiment reagent used are as follows: Ether, methanol, 75% ethanol, 95% ethanol and absolute ethyl alcohol (Hangzhou Chemical Reagent Co., Ltd., Zhejiang, China); DMEM high glucose medium, PBS, 0.25% trypsin -EDTA, penicillin and streptomycin (Hangzhou Gino Biological Pharmaceutical Co., Ltd., Zhejiang, China); FBS(Gibco corporation, New York, USA); MTT (Sigma-Aldrich, USA); DAPI (Roche Ltd, Shanghai, China); rabbit anti-human P21, P27, MMP-2, MMP-9 polyclonal antibody(Abcam, Burlingame, CA, USA); rabbit anti-human AKT, p-AKT polyclonal antibody (Cell Signaling Technology, Inc, USA); horseradish peroxidase-labeled goat anti-rabbit or anti-mouse secondary antibody, FITC, FRITC labeled goat anti-rabbit IgG(Jackson Immuno Research Laboratories, Inc, USA); Western blot and zymography related Reagents (Beyotime Biotechnology Institute, Jiangsu, China); anti-β-actin (Sigma-Aldrich Co., USA) .

The article "Lycium barbarum polysaccharides inhibit proliferation and migration of bladder cancer cell lines BIU87 by suppressing Pi3K/AKT pathway" was retracted in 2026. Reasons: plagiarized images; duplicated images; overlap with other authors' work; original data or images not available.

### Cell culture

Human bladder cancer cell lines BIU87 was purchased from Shanghai Bioleaf Co., Ltd. (Shanghai, China). Cells were cultured at 37°C with 5% CO_2_ humidified atmosphere, in DMEM supplemented with 10% FBS and 1% penicillin/streptomycin.

### RNA isolation and qRT-PCR

Total RNA of cell lysates was extracted in accordance with TRIzol solution (Invitrogen Life Technologies, Carlsbad, CA, USA). 2 μg of RNA was taken to synthesize cDNA using M-MLV Reversereverse transcription reaction system (Invitrogen). oligo (deoxythymidine)_20_ was used as primers.

Quantitative real-time PCR was conducted using BioRad Real-Time PCR detection system, using SYBR (Roche). Relative expression levels were determined using 2^−ΔΔCt^ methods. GAPDH was applied as the internal control and amplified. The amplification protocol included denaturation at 95°C for 1 min, annealing at 60°C for 10 sec, extension at 72°C for 30 sec for 35 cycles. All the experiments were performed for three times.

### MTT analysis

MTT assay was performed to measure proliferation of BIU87 cells. BIU87 cells (6000 per well) were placed in 96-well plates. After the cells had been adherented, they were cultured in serum-free medium for 24 h to be synchronize. The intervention factor corresponding to each category was added to each group with three repeated wells and two blank wells without cells in each group. Cells were cultured for 24 h, 48 h and 72 h under respective condition. After cultured, each well was added with 20 μL of MTT (3-(4, 5-dimethylthiazol-2-yl)-2, 5-diphenyltetrazolium bromide). The treated cells were further incubated for 4 hours under 37°C. The culture medium was removed and each well had with 150 μl of dimethylsulfoxide. Then cells were shocked for 10 minutes. Absorbance was read on an ELISA plate reader at 570 nm. Each assay was done in triplicate and the result was taken as the average of three. Cell growth curve of BIU87 was plotted with time as the horizontal axis and absorbance as the vertical axis.

### Cell cycle analysis

The effect of LBP on cell cycle distribution was measured by flow cytometry. Briefly, 2 × 10^5^ cells were seeded into the 12-plates and allowed to attach overnight. Cells were dealt with 400, 800 and 1200 μg/ml of LBP. 48 hours later, cells were harvested and centrifuged for 5 min at 2000 rpm. Then cells were washed by PBS and fixed using 70% ethanol at 4°C overnight. The cells were incubated with 100 mg/ml RNase for 30 min and collected with FACSort flow cytometer. The data were analyzed with FlowJo7.6.

The article "Lycium barbarum polysaccharides inhibit proliferation and migration of bladder cancer cell lines BIU87 by suppressing Pi3K/AKT pathway" was retracted in 2026. Reasons: plagiarized images; duplicated images; overlap with other authors' work; original data or images not available.

### Wound healing

2 × 10^6^ cells per well were seeded in 6-well plates and cultured for approximately 24 hours to be nearly confluent. A p200 pipette tip was used to make the scratch “wound”, the FBS free medium was changed to remove detached cells. The cells were cultured under the same conditions. Photoes at 0,12,24,48 and 72 hour were taken. Cell migration area was calculated by image pro plus6.0 software (the formerly scratch area minus the final vacant area between cells). The ratio of migration area to the formerly scratch area indicates how many BIU87 cells migrate.

### Transwell assay

5 × 10^4^ cells in each group were washed with PBS and seeded on the top of BD Matrigel™ Invasion Chambers without serum, according to the manufacturer's introductions. 10% fetal bovine serum media was placed in the lower chamber. After allowed to invade for 10 hours, cell invasion was assessed by counting the cells that migrated to the bottom of the chamber using crystal violet staining. 5 random fields per well for each replicate.

### Western blot (WB)

Cells were collected and lysed in SDS lysis buffer. Followed by centrifugation and heated at 95°C for 10 min the protein was resolved by 10% sodium dodecyl sulfatepolyacrylamide gel electrophoresis (SDS-PAGE), following transferred onto nitrocellulose membrane. The membrane was bolcked with 5% non-fat milk in Tris-buffered saline (PBS) containing Tween 20 (0.05%). The membrane was incubated with the primary antibody at 4°C overnight, following incubated with horseradish peroxidase-conjugated goat anti-rabbit secondary antibody or goat anti-mouse secondary antibody for 1 hour. Finally, the immunoreactive bands were visualized with the enhanced chemiluminescence system.

### Statistical analysis

Data was presented as the means ± SD. All experiments were performed at least three times. Statistical analysis for multiple groups was evaluated by One-way ANOVA and LSD method. *P* < 0.05 was considered as significant. Statistical Package for Social Scientists (SPSS, version 18.0, IL) was used for all analyses.
